This article has been retracted.

# Impacts of Ultrasound-Guided Nerve Block Combined with General Anesthesia with Laryngeal Mask on the Patients with Lower Extremity Fractures

**DOI:** 10.1155/2022/3603949

**Published:** 2022-09-20

**Authors:** Xiaoxu Yang, Lei Bao, Xue Gong, Hui Zhong

**Affiliations:** Anesthesia Operation Center, Chengdu Seventh People's Hospital, China

## Abstract

**Objective:**

Surgical reduction is the leading approach to patients with lower extremity fractures. The options of anesthetic drugs during surgery are of great significance to postoperative recovery of patients. There is no consensus on the optimum anesthesia method for patients undergoing lower extremity fracture surgery. Our study is aimed at investigating the impacts of nerve block combined with general anesthesia on perioperative outcomes of the patients.

**Methods:**

In this retrospective study, 48 patients experienced general anesthesia only, and 42 patients received never block combined with general anesthesia. The perioperative hemodynamics was recorded, including mean arterial pressure (MAP), oxygen saturation of blood (SpO2), and heart rate (HR). Visual analogue scale (VAS) and Montreal Cognitive Assessment (MoCA) were carried out to evaluate postoperative pain and cognitive status. Furthermore, adverse reactions and recovery condition were observed between the patients receiving different anesthesia methods.

**Results:**

At 15 minutes and 30 minutes after anesthesia, as well as 5 minutes after surgery, significant lower MAP was observed in the patients treated with general anesthesia (83.04 ± 8.661, 79.17 ± 9.427, 86.58 ± 8.913) compared to those receiving never block combined with general anesthesia (90.43 ± 4.618, 88.74 ± 6.224, 92.21 ± 4.015) (*P* < 0.05), and compared with general anesthesia group (68.5 ± 7.05, 69.63 ± 7.956, 72.75 ± 8.446), the combined anesthesia group (73.52 ± 9.451, 74.17 ± 10.13, 77.62 ± 9.768) showed obvious higher HR (*P* < 0.05). No significant difference in SpO_2_ was found between the two groups at multiple time points (*P* > 0.05). As for the score of VAS and MoCA, remarkably lower VAS and higher MoCA at 6 h, 12 h and 24 h after surgery were presented in the combined anesthesia group compared to general anesthesia group (*P* < 0.05). At 24 h after surgery, the two groups showed normal cognitive function (26.33 ± 0.7244 vs. 28.55 ± 0.7392). Incidence of nausea and vomiting in the combined anesthesia group was lower than that of the general anesthesia group (*P* < 0.05). The time to out-of-bed activity and hospital stay were shorter in the combined anesthesia group compared with general anesthesia (*P* < 0.05).

**Conclusion:**

The application of never block combined with general anesthesia contributed to the stability of hemodynamics, alleviation of postoperative pain and cognitive impairment, along with decrease in adverse reactions and hospital stay in the patients with lower extremity fractures.

## 1. Introduction

Age induced bone loss increases the risk of lower extremity fracture in the middle-aged and elderly populations [1, 2]. Approximately 33% of adult women and 50% of adult men suffered from extremity fracture before the age of 65 [3]. Lower extremity fracture has been reported to pose an escalating burden on public health care and result in long-term adverse effects on the quality of life of patients, such as impairments or loss of physical function [4]. Lower extremity fracture, as a prevalent type of fracture in clinic, is generally treated with surgical reduction, which is common in orthopedic surgery. The operation time of lower extremity fracture is relative long, which has a significant impact on the patient's respiratory and circulatory system [5]. In addition, the patients tend to experience acute pain during postoperative period as a result of large-scale traumatic injury, leading to an adverse impact on postoperative functional exercise [6]. Therefore, an appropriate anesthesia program is of great significance in reducing the occurrence of stress reaction and complications, and accelerating the postoperative rehabilitation of patients.

General anesthesia is a common anesthesia method in lower extremity fracture surgery, but it's a challenging for the physiology and postoperative rehabilitation of elderly patients [7, 8]. Comparing with general anesthesia, ultrasound-guided nerve block has special advantages such as relatively high safety and physiological interference reduction. With the help of ultrasound guidance, nerve block can accurately locate the anesthesia site and clarify the paths of drug diffusion, which may end up with optimal anesthesia effect and decrease in unnecessary injury. In recent years, ultrasound-guided nerve block is increasingly used in fracture surgery, especially in elderly patients [9–11]. However, as described in previous studies, nerve block might lead to block failure or incomplete block. For instance, the failure rate of fascia iliaca compartment block used to block the lateral femoral cutaneous nerve is 10% - 37% [12]. 3 of 78 patients failed to receive lumbosacral nerve root block and 75 patients showed tapping sensation at L5 region without contraction of muscles [13]. Enhanced recovery after surgery (ERAS) is a combination of multimodal evidence-based strategies that has been proved to be an effective treatment for perioperative patient care in various diseases including fracture. It can reduce perioperative stress reaction of patients, shorten hospital stay, and decrease the incidence of postoperative complications and mortality, thus accelerating postoperative recovery of patients [14, 15]. On the basis of the concept of ERAS, combined anesthesia has been widely applied to a variety of surgeries, such as off-pump coronary artery bypass graft surgery [16] and hip replacement surgery [17]. It is well established that ultrasound-guided nerve block combined with additional intravenous anesthetic drugs contribute to improvement of the anesthetic effect in intertrochanteric fracture [18] and unilateral rib fracture [19].

In our study, we enrolled 90 patients undergoing lower extremity fracture surgery and divided them into two groups according to anesthesia scheme. Among them, 48 patients received general anesthesia alone, and the remaining patients underwent nerve block combined with general anesthesia. The purpose of this study was to explore the effects of nerve block combined with general anesthesia in patients with lower extremity fracture.

## 2. Materials and Methods

### 2.1. Study Population

A total of 90 patients undergoing lower extremity fracture surgery in our hospital from December 2019 to June 2021 were enrolled in this retrospective study. During the surgery, 48 patients experienced general anesthesia (general anesthesia group), consisting of 28 males and 20 females, who were 18-65 years of age (49.67 ± 3.21 mean age). The remaining 42 patients aged 18 to 64 years (50.32 ± 2.98 mean age), including 25 males and 17 females, received nerve block combined with general anesthesia (combined anesthesia group) based on the concept of ERAS. The body mass of general anesthesia group and combined anesthesia group was 58.5 ± 2.3 vs. 57.8 ± 2.6. In the general anesthesia group, there were 32 cases and 16 cases with class I and II of the American Association of Anesthesiologists (ASA), respectively. 28 and 14 of patients in the combined anesthesia group presented ASA class I and II, respectively. The operation time of general anesthesia group and combined anesthesia group was 65-85 min (72.28 ± 4.64) and 63-84 min (73.34 ± 5.14), respectively. Comparing the baseline data of the two groups, the difference was not statistically significant (Supplementary table 1, *P* > 0.05). All eligible patients were known to be diagnosed with American Society of Anesthesiologists (ASA) class I-II lower extremity fractures by imaging examinations such as CT and X-ray and presented complete clinical data. Those diagnosed patients with cognitive impairment, abnormal coagulation function, and contraindications of surgery and anesthesia, as well as dysfunction of multiple organs, were excluded in the study. The study was approved by the ethics committee of our hospital, and obtained signed written informed consent form from each included patient.

### 2.2. Approaches of Anesthesia

All patients received health education and psychological guidance after admission. 300 ml of 5% glucose was taken orally 2 hours before operation. Hemodynamic monitoring including mean arterial pressure (MAP), oxygen saturation of blood (SpO_2_), and heart rate (HR) was performed before anesthesia. Furthermore, the peripheral venous access of the nonoperative upper limb was established and compound sodium chloride was infused (10 ml/kg/h). Dexmedetomidine (1.0 ug/kg) was injected intravenously 15 minutes before anesthesia to alleviate preoperative anxiety and pain caused by body position changing during anesthesia operation. The general anesthesia group was treated with intravenous injection of fentanyl citrate (drug approval number: H42022076) (5 *μ*g/kg) and propofol (drug approval number: H20051842) (2 mg/kg), and cisatracurium besilate (drug approval number: H20090202) (0.2 mg/kg), successively. 3 minutes of mask controlled ventilation was conducted after the decrease of eyelash reflex, followed by oxygen inhalation through laryngeal mask, with ventilator parameter of tidal volume (TV) 8-10 ml/kg and respiratory rate (RR) 10-12 times/min. Inhalation of 2%~3% sevoflurane (drug approval number: H20070172) was used to maintain intraoperative anesthesia, and additional of fentanyl citrate and cisatracurium besilate was adopted as required. The parameter of end-tidal CO_2_ pressure (PETCO_2_) and bispectral index (BIS) was maintained 35-45 mmHg and 40-50, respectively.

The combined anesthesia group received nerve block combined with general anesthesia. Ultrasound-guided nerve block anesthesia of the affected limb was first applied to the patients with supine position. A portable ultrasonic instrument (frequency 6-13 Hz) was used to locate the femoral artery, femoral vein, and femoral nerve of the patient for performance of fascia iliaca compartment block. In brief, 25 ml of 0.5% ropivacaine mesylate (drug approval number: H20051865) as local anesthesia was implemented following punctured iliac fascia by the needle, and then the patients, who were kept in position of elevated hip and bended knee of the affected side, underwent sciatic nerve block under ultrasound. The needle was punctured into sciatic nerve after trochanter was located by ultrasound, followed by local anesthesia injection with 15 ml of 0.5% ropivacaine mesylate. The blocking effect was detected by acupuncture, which followed the complete performance of sciatic nerve block. The sensory and motor block was measured every 5 minutes, and those patients should be excluded from the study if blocking failure happened to them within 30 minutes. Intravenous general anesthesia was carried out after confirmation of the block effect. The patients were given injection of fentanyl citrate (1 *μ*g/kg) and propofol (2-2.5 mg/kg) and received 3 minutes of oxygen inhalation via mask after eyelash reflex was weakened. Inhalation of 2%~3% sevoflurane was performed after installation of laryngeal mask. During the operation, the patient was maintained spontaneous breathing. Fentanyl (0.05-0.1 mg) was added once if RR was more than 20 times/min, and manual or mechanical ventilation (PETCO_2:_ 35-55mmHg, SpO_2_ > 97%) was given in the case of insufficient respiratory ventilation. During surgery, if the decrease of MAP of patients was more than 20% of the basic value, ephedrine (3 mg/time) or phenylephedrine (0.01 mg/time) shall be given. Fentanyl (0.05-0.1 mg/time) was applied to the patients with MAP elevation more than 20% of the basic value and HR increase exceeding 10% of the basic value. The patients with HR < 50 beats/min should be treated with atropine (0.2 mg/time). The laryngeal mask was removed when the patient was fully awake after the operation.

### 2.3. Postoperative Analgesia

All patients were transferred to postanesthesia care unit (PACU) and received intravenous infusion of 8 mg of ondansetron (drug approval number: H10970065) after operation. Postoperative patient-controlled intravenous analgesia (PCIA) with 0.8 mg of fentanyl diluted to 100 ml by normal saline was used for postoperative pain alleviation within 48 hours. The loading dose of the first intravenous injection was 5 ml, and the predesigned infusion rate was 2 ml/h. Dose of PCIA was set to 2 ml/time, and 15 minutes were regarded as the lockout time.

### 2.4. Outcome Evaluation

Hemodynamics variables, including MAP, HR, and SpO_2,_ were monitored and recorded in the two groups before anesthesia, 15 minutes after anesthesia, 30 minutes after anesthesia, and 5 minutes after surgery.

Visual analogue scale (VAS) [20] was used to evaluate the pain intensity of patients at 6 h, 12 h, and 24 h after surgery. VAS score ranges from 0 to 10, and the scores are positively correlated with pain intensity. In general, no pain is described by 0 scores. 1-3 scores are regarded as mild pain, 4-6 scores indicates moderate pain, and 7-10 scores present severe pain. Postoperative cognitive status was assessed using Montreal Cognitive Assessment (MoCA) [21] . The scale includes 8 dimensions, including attention and concentration, orientation, executive function, abstract thinking, language, memory, visual structure skills, and calculation. There are 11 scoring items in total, with a total score of 30. The higher the score is, the higher the cognitive function. Generally, cognitive function is normal with a score greater than or equal to 26, the score of mild cognitive impairment and moderate cognitive impairment is between 18 and 26, and 10 and 17, respectively. The scores lower than 10 are regarded as severe cognitive impairment.

The adverse reactions of patients in the two groups receiving different anesthesia were observed after surgery, including dizziness and headache, nausea and vomiting, drowsiness, urinary retention, and respiratory depression.

### 2.5. Statistical Analysis

SPSS 22.0 software was adopted for data analysis. T test or F test was applied to analyze measurement data described as mean ± standard deviation. The counting data were expressed as percentage (%) and determined by Chi-square test. *P* < 0.05 indicated that the difference was statistically significant.

## 3. Results

### 3.1. Hemodynamic Variables of the Two Groups at Multiple Time Points

The patients in the two groups showed no significant difference in terms of MAP, HR, and SpO_2_ before anesthesia (*P* > 0.05). At 15 minutes after anesthesia and 30 minutes after anesthesia, MAP was decreased in the two groups, and the patients treated with general anesthesia had lower MAP than the patients undergoing nerve block combined with general anesthesia (*P* < 0.05). MAP was increased at 5 minutes after surgery in both two groups, and higher MAP was showed in the combined anesthesia group compared to general anesthesia group (*P* < 0.05). As for changes of HR, the two groups exhibited declined HR at 15 minutes after anesthesia, and the downward trend was more obvious in general anesthesia group (*P* < 0.05). At 30 minutes after anesthesia and 5 minutes after surgery, more elevated HR was observed in the patients receiving nerve block combined with general anesthesia compared to those who were given general anesthesia (*P* < 0.05). However, there was no significant different in SpO_2_ between the two groups at multiple time points (*P* > 0.05, Table 1).

### 3.2. Alleviation of Postoperative Pain by General Anesthesia Combined with Nerve Block

VAS was performed to assess the postoperative pain in both groups. As listed in Table 2, combined anesthesia group and general anesthesia group exhibited the strongest pain intensity at 6 h after surgery (3.548 ± 0.5038 vs. 4.667 ± 0.5955, *P* < 0.05), and the VAS score in the two groups at 12 and 24 h after surgery was lower than that at 6 hours after surgery (*P* < 0.05). Furthermore, VAS score of combined anesthesia group at 12 h and 24 h after surgery was 2.571 ± 1.129 and 1.952 ± 1.229, respectively, which was significant lower than that of general anesthesia group (3.708 ± 1.051, 3.063 ± 1.21) (*P* < 0.05).

### 3.3. Reduced Cognitive Impairment by General Anesthesia Combined with Nerve Block

MoCA was applied to evaluate cognitive status of all patients during perioperative period. The MoCA score before surgery was not significant different between combined anesthesia group and general anesthesia group (*P* > 0.05), with normal cognitive function (28.43 ± 0.8007 vs. 28.35 ± 0.5645). The MoCA score of general anesthesia group and combined anesthesia group was 23.4 ± 0.7646 and 26.69 ± 0.4679 at 6 h after surgery, which was obviously lower than that before surgery (*P* < 0.05). In addition, at 12 h and 24 h after surgery, the two groups both showed elevated MoCA score, and the patients undergoing nerve block combined with general anesthesia presented much higher score than those receiving general anesthesia (*P* < 0.05, Table 3).

### 3.4. The Postoperative Adverse Reactions and Recovery Condition of the Two Groups

Adverse reactions were observed and compared between the two groups, including dizziness and headache, nausea and vomiting, drowsiness, urinary retention, and respiratory depression. As shown in Table 4, we found that the incidence of nausea and vomiting was 25% and 7.14% in general anesthesia group and combined anesthesia group (*P* < 0.05). Although lower incidence of dizziness and headache, drowsiness, and urinary retention was found in combined anesthesia group compared to general anesthesia group, the difference was not significant (*P* > 0.05). No patients suffered from respiratory depression in both groups, and the patients in general anesthesia group showed higher total incidence of adverse reactions than those in combined anesthesia group (*P* < 0.05). Furthermore, we observed that the time to out-of-bed activity and hospital stay of the patients receiving combined anesthesia were significantly shorter than that of patients only undergoing general anesthesia (*P* < 0.05).

## 4. Discussion

Surgical reduction is the main treatment for lower extremity fracture. Various factors during the perioperative period, including trauma, blood loss, pain, changes in total circulation, and emotional tension, result in strong stress response in the patients. In addition, postoperative swelling of affected limbs, incision pain, and strong stimulation of nerves at the fracture site exacerbated the acute pain after surgery. Approximately 25%-35% of the patients suffered from postoperative pain, which affected physical function of the affected limb and negatively affected the postoperative rehabilitation [22]. Therefore, attention should be paid to the design of anesthesia scheme in the operation of lower extremity fracture.

In the past, epidural block anesthesia was widely used in patients undergoing lower extremity surgery due to its advantages of good anesthetic effect. However, it is not applicable to those patients with spinal ligament calcification or intervertebral space stenosis [23]. Furthermore, the respiratory and circulatory systems of some patients will also be affected [24]. In contrast, general anesthesia is more convenient for anesthesia management of patients, but it will affect the stability of hemodynamics of patients. Therefore, it is often combined with nerve block in clinic to improve postoperative outcomes in fracture surgery [19, 25, 26]. In our retrospective study, we analyzed the impacts of general anesthesia and nerve block combined with general anesthesia in patients undergoing lower extremity fracture. We monitored the hemodynamic changes between the two groups at multiple time points and found that MAP at 15 minutes and 30 minutes after anesthesia, as well as 5 minutes after surgery in the two groups was lower than that of before anesthesia, respectively. Comparing to the general anesthesia group, the combined anesthesia group presented obvious higher MAP at multiple time points except for before anesthesia (*P* < 0.05). Furthermore, more stable MAP was revealed in the combined anesthesia group compared with the general anesthesia group (95.33 ± 3.545, 90.43 ± 4.618, 88.74 ± 6.224, 92.21 ± 4.015) vs. (94.56 ± 4.136, 83.04 ± 8.661, 79.17 ± 9.427, 86.58 ± 8.913). No significant difference in HR before anesthesia was found between the general anesthesia group (77 ± 8.495) and combined anesthesia group (76.48 ± 9.195). However, at 15 minutes and 30 minutes after anesthesia, along with 5 minutes after surgery, the combined anesthesia group had higher HR when it was compared with general anesthesia group (*P* < 0.05). As for SpO_2_ variables, there was no significant different between the two groups at multiple time points (*P* > 0.05). As reported in previous studies [18], Liu et al. indicated that compared with the combined spinal-epidural anesthesia, the general anesthesia with laryngeal mask airway and nerve block contributed to slight intraoperative hemodynamic variations of the elderly patients with intertrochanteric fracture surgery. In the hip surgery, significant reductions in MAP at induction was observed in the patients treated with general anesthesia compared to those undergoing general anesthesia combined with nerve block. Besides that, block group presented no significant changes in cardiac output, cardiac index, stroke volume, and stroke volume index [27]. Peripheral nerve block damages the conduction of noxious stimulation and significantly reduces stress response. A large number of studies have confirmed that nerve block effectively optimizes perioperative analgesia and reduces the use of intraoperative and postoperative analgesics [28–30]. However, the locations where nerve block can be performed are relatively limited. A certain dose of additional intravenous sedatives or general anesthesia is required to obtain the best anesthetic effect, resulting in guarantee of adequate oxygen supply during surgery. A study of total knee arthroplasty demonstrated that femoral nerve block combined with general anesthesia alleviated postoperative pain and exhibited declined 6 h and 24 h VAS scores in resting state after surgery [31]. In the present study, comparing to general anesthesia group, the combined anesthesia group had much lower VAS score at 6 h, 12 h, and 24 h after surgery. We also found that the patients receiving nerve block combined with general anesthesia showed higher MoCA score at postoperative multiple time points Ultrasound-guided nerve block is associated with improvement in the controllability of anesthetic dispersion and reduction in the damage to peripheral nerves and blood vessels. It leads to little effect on patients' cognitive function. As reported by total knee arthroplasty study, the rate of postoperative cognitive dysfunction at 4 d and VAS scores at 4-48 h after surgery was lower in the group receiving ultrasound-guided femoral nerve block in contrast to the group undergoing intravenous infusions of fentanyl [32]. Our study compared the postoperative adverse reactions between the two groups. The incidence of nausea and vomiting was 25% and 7.14% in general anesthesia group and combined anesthesia group, respectively. No remarkable difference was observed in terms of incidence of dizziness and headache, drowsiness, and urinary retention between the two groups. The increase in the incidence of nausea and vomiting might be related to the excessive use of general anesthesia drugs. Opioids cause gastrointestinal peristalsis to slow down by activating U-type opioid receptors distributed in the presynaptic nerve endings of the intestinal muscle plexus. At the same time, opioid receptor causes central reaction, leading to nausea and vomiting [33]. Furthermore, nerve block combined with general anesthesia is conductive to early recovery, which was presented by short time to out-of-bed activity and hospital stay.

In conclusion, ultrasound-guided nerve block combined with general anesthesia contributed to maintaining the stability of hemodynamics and alleviating cognitive impairment. Furthermore, it is conducive to relief of postoperative pain, resulting in early recovery of lower extremity function. However, some limitations existed in this study, including lack of follow-up data and analysis of pain related inflammatory response. Besides, in the future, larger clinical samples of lower extremity fractures are needed to verify and refine our results.

## Figures and Tables

**Table 1:** Hemodynamics variables of the two groups at multiple time points.

Group	*N*	MAP(mmHg)				HR (beats/minute)				SPO2 (%)			
		Before anesthesia	15 minutes after anesthesia	30 minutes after anesthesia	5 minutes after surgery	Before anesthesia	15 minutes after anesthesia	30 minutes after anesthesia	5 minutes after surgery	Before anesthesia	15 minutes after anesthesia	30 minutes after anesthesia	5 minutes after surgery
General anesthesia	48	94.56 ± 4.136	83.04 ± 8.661	79.17 ± 9.427	86.58 ± 8.913	77 ± 8.495	68.5 ± 7.05	69.63 ± 7.956	72.75 ± 8.446	97.35 ± 1.329	97.23 ± 1.491	96.88 ± 1.817	96.98 ± 1.591
Combined anesthesia	42	95.33 ± 3.545	90.43 ± 4.618	88.74 ± 6.224	92.21 ± 4.015	76.48 ± 9.195	73.52 ± 9.451	74.17 ± 10.13	77.62 ± 9.768	97.14 ± 1.69	97.31 ± 1.76	97 ± 1.9	97.29 ± 1.715
*t*		0.9423	4.944	5.597	3.771	0.2808	2.88	2.379	2.536	0.6632	0.2345	0.3187	0.8794
*P*		0.3486	< 0.0001	< 0.0001	0.0003	0.7795	0.005	0.0195	0.013	0.5089	0.8151	0.7507	0.3816

**Table 2:** VAS score for evaluation of postoperative pain.

Group	*N*	6 h after surgery	12 h after surgery	24 h after surgery	*F*	*P*
General anesthesia	48	4.667 ± 0.5955	3.708 ± 1.051	3.063 ± 1.21	32.09	< 0.0001
Combined anesthesia	42	3.548 ± 0.5038	2.571 ± 1.129	1.952 ± 1.229	26.82	< 0.0001
*t*		9.549	4.945	4.311		
*P*		< 0.0001	< 0.0001	< 0.001		

**Table 3:** MoCA score for assessment of perioperative cognitive function.

Group	*N*	Before surgery	6 h after surgery	12 h after surgery	24 h after surgery	*F*	*P*
General anesthesia	48	28.35 ± 0.5645	23.4 ± 0.7646	24.54 ± 0.5035	26.33 ± 0.7244	536.2	< 0.0001
Combined anesthesia	42	28.43 ± 0.8007	26.69 ± 0.4679	27.93 ± 1.113	28.55 ± 0.7392	45.78	< 0.0001
*t*		0.5143	24.23	18.99	14.33		
*P*		0.6084	< 0.0001	< 0.0001	< 0.0001		

**Table 4:** Incidence of postoperative adverse reactions (*n*, %) and recovery condition in the two groups.

Group	Nausea and vomiting	Dizziness and headache	Drowsiness	Urinary retention	Respiratory depression	Total adverse reactions	Time to out-of-bed activity (h)	Hospital stay (d)
General anesthesia	12 (25)	2 (4.17)	5 (10.42)	3 (6.25)	0 (0)	22 (45.83)	42.18 ± 4.4323	11.9 ± 0.9579
Combined anesthesia	3 (7.14)	0 (0)	1 (2.38)	2 (4.76)	0 (0)	6 (14.29)	30.09 ± 4.3782	7.79 ± 0.9762
*Chi-square*	5.143	1.79	2.325	0.09454	/	10.4		
*t*	/	/	/	/	/	/	12.98	20.13
*P*	0.0233	0.181	0.1273	0.7585	/	0.0013	< 0.0001	< 0.0001

## Data Availability

The data used to support the findings are in the article.

## Supplementary Materials

Supplementary Materials Baseline data of the two groups.
